# Assessment and Discussion of Correlation Among Psychological Symptoms, Occupational Strain, and Neurotic Personality for Metro Drive

**DOI:** 10.3389/fpsyg.2022.823682

**Published:** 2022-05-16

**Authors:** Jing He, Yanling Zhang, Si Qin, Wei Liu

**Affiliations:** ^1^Faculty of Transportation Engineering, Kunming University of Science and Technology, Kunming, China; ^2^Yunnan University of Business Management, Kunming, China; ^3^Kunming Rail Transit Operation Co., Ltd., Kunming, China

**Keywords:** metro driver, psychological symptom, neuroticism, occupational strain, mediating role

## Abstract

Metro driver is the prime person who is responsible for metro operation safety. The mental health of a metro driver is very important for the operation of the subway and requires the driver to keep high mental alertness to monitor the surrounding environment and also handle emergencies under uncertain or dangerous conditions. After a long-term occupational strain, a metro driver is likely to suffer from some mental health problems, such as anxiety and depression, that ultimately threaten the lives of passengers. Therefore, in this study, we focus on the psychological symptoms of metro drivers from the angle of occupational strain and neuroticism. A total of 396 metro drivers from Kunming Rail Transit Operation Co., Ltd. in China were investigated through a questionnaire survey. Symptom Checklist-90 (SCL-90), Personal Strain Questionnaire (PSQ), and NEO-Five-Factor Inventory-Neuroticism Subscale (NEO-FFI-N) were applied to evaluate the psychological symptoms, occupational strain, and neuroticism in metro drivers, respectively. The surveyed data were analyzed by SPSS software. Based on the data, a path structural equation model was established to explore the correlation among occupational strain, psychological symptoms, and neuroticism. The results show that the scores for psychological symptoms and occupational strain are higher than the Chinese adult norm among metro drivers. The occupational strain, neuroticism, and psychological symptoms are all positively correlated in the metro drivers. Occupational stress has a direct influence on the psychological symptom, while neuroticism plays a partial mediation role between occupational strain and psychological symptoms. The results of this study can be applied to optimize the employee selection system and training system for metro operation companies.

## Introduction

Subway train operation is a complex and socio-technical system that requires the metro driver to keep high mental alertness to monitor the surrounding environment and also handle emergencies instantaneously under dangerous conditions. In such a high-intensive and persistent job environment, metro drivers not only endure the pressure related to the job, but also need to overcome the fatigue and languor caused by high-intensive work. Therefore, after working for a long term, chronic mental stress will produce a negative impact on the physical and mental health of metro drivers. In addition, the subway train operation not only requires that the metro driver has a good professional quality to realize the modernization operation, but also requires the metro driver to bear the repetitive dry operation and boring working environment which will undoubtedly lead to the occurrence of adverse psychological symptoms among the metro drivers. With the improvement of automation, the errors caused by machines rarely occur in subway operations. On the contrary, human operation error has gradually become the main cause of driving accidents, and most of the accidents are caused by the unsafe behavior of humans, which is further related to psychological factors. Therefore, the mental health of metro drivers directly affects the safety of thousands of passengers and the service quality of trains.

Many studies have focused on transportation accidents and analyzing the causes of the accident (Wang et al., 2014; Fan et al., 2015; Garcia-Herrero et al., 2021; Zhai et al., 2021). Most results showed that more than 80% of accidents are caused by driver’s operation error, and 90% of accidents are related to the driver’s response to stress conditions, which is influenced by a driver’s anxiety, depression, and other psychological diseases. In a previous study (Hlotova et al., 2014), the authors studied the psychological symptoms among bus drivers and found that the bus driving job is one of the most stressful occupations, with 97% of the bus drivers having an occupational strain. In other studies (Chung and Wu, 2013; Fındık et al., 2018), the authors found that individual occupational strain could produce professional burnout and further threaten driving safety. In one study (Lee et al., 2014), the authors found that occupational strain is one of the most important factors that can cause psychological problems among metro drivers. The metro driver is required to possess certain special professional skills, which necessitate that the driver not only possess a strong responsibility and safety awareness, but should also have proficient train operation and fault disposal skills under abnormal conditions. Therefore, it is highly important to study the relationship between occupational strain and psychological symptoms among metro drivers to improve their psychological health and eventually promote the safety of subway operations.

Some studies have also found that personality also has a significant influence on driving safety. In previous studies (Vittengl, 2017; Sosnowska et al., 2019), the authors demonstrated that the traffic accidents caused by drivers with neuroticism are 80% higher than those caused by drivers without neuroticism, as the drivers with neuroticism are more prone to be affected by the negative psychological symptoms, such as anxiety, compulsion, and hostility, under high-pressure working conditions. Some authors further found that there is a certain correlation between neuroticism and traffic accidents (Bergomi et al., 2017; Wang et al., 2018; Mamcarz et al., 2019; Ye et al., 2021). Some researchers (Guo et al., 2016) found that neuroticism is an important factor that can be used to predict dangerous driving behavior (Shen et al., 2013; Jin et al., 2019). The living environment has a significant impact on personality development, which can be cultivated and changed in the living environment. An individual under long-term occupational strain has an increased tendency to develop neuroticism, which can subsequently lead to some mental health problems, such as anxiety and depression. Therefore, there is a definite relationship among occupational strain, neuroticism, and psychological symptoms.

Through literature analysis, it has been found that occupational strain and neuroticism can affect individual psychological symptoms, and high occupational strain can lead to neuroticism (Gabriela et al., 2020). Therefore, there is a certain correlation between occupational strain, neuroticism, and psychological symptoms. Therefore, in this study, to evaluate the mental health of the metro driver, the psychological symptoms, occupational strain, and personality of the metro driver are investigated to determine the correlation among the occupational strain, neuroticism, and psychological symptoms. The important contributions of this research are in three areas: (1) a path structural equation model (SEM) is established to analyze the relationship among occupational strain, psychological symptoms, and neuroticism; (2) this study finds that neuroticism plays a significant mediating role between occupational strain and psychological symptom; and (3) the results of the study can provide a theoretical foundation for the metro operating companies to optimize metro driver workflow, evaluate driver performance, and formulate recruitment principles.

The rest of this paper is organized as follows: Section II provides details about the study subjects, tools used, and statistical methods. Section III addresses the data analysis results. Section IV presents the results and discussion. Finally, Section V includes the conclusion and summary.

## Materials and Methods

### Study Subjects

In this study, a total of 417 on-the-job metro drivers from Kunming Rail Operation Co., Ltd. in Yunnan Province of China were selected to conduct a questionnaire survey and collect data regarding occupational strain, psychological symptoms, and neuroticism. The questionnaire survey was approved by Kunming Rail Transit Operation Co., Ltd. Since Kunming Rail Transit Operation Co., Ltd. does not have an established ethics review committee at present, all the research procedures were approved by the company. Prior to the survey, the metro drivers with mental illness or other brain organic lesions were eliminated through their personal records and annual physical examination reports from the company. Before the survey, the metro drivers were informed about the following conditions: (1) If they decided to participate in this survey, their personal information would be kept confidential and the information will be accessible only to them; (2) when the survey results are published, their personal information will be not disclosed; and (3) all on-the-job metro drivers need to sign an informed consent form. The survey was conducted from April 2021 to July 2021. All methods were performed in accordance with relevant guidelines and regulations that include Revised Declaration of Association Medical Mondiale (2013), Urban Rail Transit Operation Management Regulations, Interim Measures for Safety Assessment and Management before and during the Official Operation of Urban Rail Transportation and Technical Specifications for Pre-operation Safety Assessment of Urban Rail Transit Part 1: Metro and Light Rail. Inclusion criteria were as follows: (1) in-service metro drivers with an age range of 18–45 years; (2) working age > 1 year; (3) no organic lesions in the brain; (4) no history of mental illness; (5) and no obstacle to filling out the questionnaire independently.

After the survey, 21 invalid questionnaires were excluded, and 396 valid questionnaires were recovered with an effective rate of 94.96%. The data were analyzed based on the statistical parameters of the interviewees. All the 396 metro drivers included in the study were male, with 105 being undergraduates and 204 having college degrees, 85 secondary school degrees, and two high school degrees. A total of 141 metro drivers were married, while 255 were unmarried. The mean age of drivers was 25.6 ± 3.0 years, with an age range of 19–44 years. The description of the study participants is presented in Table 1.

**TABLE 1:** Statistical description of samples.

Variable	Category	Number	Percentage
Age	18–23	83	21%
	24–26	191	48.2%
	27–30	102	25.8%
	30–45	20	5.1%
Education	High school	2	0.5%
	Secondary specialized school	85	21.5%
	Junior college	204	51.5%
	Undergraduate	105	26.5%
Position	First-class metro driver	29	7.3%
	Second-class metro driver	322	81.3%
	Foreman	45	11.4%
Marital status	Married	141	35.6%
	Unmarried	255	64.4%

#### Symptom Checklist-90

The Symptom Checklist-90 (SCL-90), proposed by Derogatis (1975), was administered to measure the psychological symptoms of metro drivers in this study. In the SCL-90, 90 problems need to be answered and include 10 dimensions: somatization (F1), compulsion (F2), interpersonal relationship (F3), depression (F4), anxiety (F5), hostility (F6), terror (F7), crankiness (F8), psychopathy (F9), and others (F10) (Wang, 1984). The SCL-90 has a wide application in the investigation of psychological health problems among different occupational groups, and the test results can reflect the mental health problems of various occupational groups from different aspects. For each question, a score of 1–5 is given: 1 = none, 2 = very light, 3 = moderate, 4 = very heavy, and 5 = severe. The higher score indicates worse mental health status, and the factor score reflects the individual symptom. In this study, the Chinese version of the SCL-90 scale was applied to evaluate the psychological health of metro drivers.

#### Personal Strain Questionnaire

The Chinese version of the Occupational Stress Inventory-Revised Edition (OSI-R) proposed by Osipow (1998) and Huang et al. (2018) was applied to investigate the occupational strain of metro drivers in this study. The test table is composed of three sub-questionnaires, namely, the Occupational Role Questionnaire (ORQ), the Personal Strain Questionnaire (PSQ), and the Personal Resources Questionnaire (PRQ). In this study, only the PSQ (comprising 40 questions) was used, and the assessment was based on four dimensions: vocational strain (VS), psychological strain (PSY), interpersonal strain (IS), and physical strain (PHS). The five-level scoring method is applied to describe the degree of stress. A high score on the questionnaire indicates severe individual stress response.

#### NEO-Five-Factor Inventory-Neuroticism Subscale

The Chinese version of the NEO-Five-Factor Inventory-Neuroticism Subscale (NEO-FFI-N) was used to measure the neuroticism among the metro drivers in this study. The test table was compiled by Costa and Mccrae (1992) and includes the following five subscales: Openness (O), Conscientiousness (C), Extraversion (E), Agreeableness (A), and Neuroticism (N) (Fortunato, 2004). The NEO-FFI-N has been widely applied in academic and clinical research of neuroticism and has good aggregation validity with other personality measurement tools (Parker and Stumpf, 1998; Kurtz and Sherker, 2003). Therefore, in this study, 12 questions were included in NEO-FFI-N to evaluate the neuroticism personality trait in metro drivers. Each question is given a score of 1–5: 1 = very disagree; 2 = basically disagree; 3 = no opinion; 4 = basically agree; and 5 = very agree.

## Results

In this study, the data obtained by questionnaire survey were analyzed using SPSS 25.0 software developed by Norman and Hadleigh (Sun and Zhou, 2019). This software has been widely applied to analyze the questionnaire data (Wiedermann and Li, 2018). In addition, to examine the mediating effect of neuroticism between occupational strain and psychological symptoms, AMOS24.0 software (developed by SPSS Corporation) was applied to construct a path structural equation model (SEM) for path analysis. Further, the Student’s *t*-test was used to evaluate whether the correlation between the psychological symptoms and occupational strain was significant among the metro drivers, and a decreasing *p*-value is an indicator of the credibility of the result that is used to evaluate the reasonability of hypothesis testing. A small *p*-value indicates reliable results. Pearson’s correlation analysis is used to measure the correlation between psychological symptoms, occupational strain, and neuroticism in metro drivers. The range of *r* is [-1, 1]. When *r* < 0, there is a linear negative correlation between the two variables. When *r* > 0, there is a linear positive correlation between the two variables. When *r* = 0, there is no obvious correlation between the two variables. Finally, an intermediary model is proposed in the study to explore the relationship between psychological symptoms, occupational strain, and neuroticism among metro drivers by combining the path analysis method and bootstrapping method.

### Reliability Analysis of Data Collected by Questionnaires

For sociology and behavioral research, it is necessary to evaluate the reliability and validity of the questionnaires by analyzing the collected data. In this study, SPSS software was applied to analyze the reliability of questionnaires. In general, Cronbach’s α coefficient is used to evaluate the reliability of questionnaires. The value of the Cronbach’s α coefficient can reflect the degree of internal consistency of questionnaires. Higher Cronbach’s α coefficient indicates a stable questionnaire structure. When the Cronbach’s α-value is below 0.6, the reliability of the questionnaire is poor. When the Cronbach’s α-value is between 0.6 and 0.7, the reliability of the questionnaire is acceptable. When the Cronbach’s α-value is greater than 0.7, the questionnaire has good reliability. In this survey, the reliability of SCL-90, PSQ, and NEO-FFI-N is presented in Table 2. It can be seen from Table 2 that the Cronbach’s α-values of the three survey questionnaires are 0.972, 0.821, and 0.701, respectively, and the values greater than 0.7 indicate that the selection of the survey scale is reasonable.

**TABLE 2:** Reliability analysis of questionnaires used in this study.

Name of questionnaire	Cronbach’s α-value
SCL-90	0.972
PSQ	0.821
NEO-FFI-N	0.701

### Validity Analysis of Questionnaires

The validity of a questionnaire refers to whether the questionnaire can accurately detect the problem being measured. However, before evaluating the validity of the questionnaire, it is necessary to test whether the questionnaire is suitable for factor analysis. In general, Kaiser–Meyer—Olykin Measure of Sampling Adequacy (KMO) and Barlett’s test of sphericity are applied to evaluate whether the questionnaire is suitable for factor analysis. When KMO < 0.7, it means that the questionnaire is not suitable for factor analysis. When 0.7 < KMO < 0.8, factor analysis can be performed. When KMO > 0.8, it means that the questionnaire is suitable for factor analysis. At the same time, when the significant probability of Barlett’s sphericity test is less than 0.05, it means that the questionnaire can be extracted by the factor method to simplify the data structure. When the KMO value and Barlett’s sphericity test for the questionnaire meet the requirements at the same time, it means that factor analysis can be performed. Table 3 gives the KMO values and Barlett’s sphericity test results of the three questionnaires. The KMO values for SCL-90, PSQ, and NEO-FFI-N are found to be 0.938, 0.897, and 0.783, respectively, and the Barlett’s sphericity test shows a significant probability of 0.000. These results indicate that the selected questionnaires are suitable for factor analysis.

**TABLE 3:** KMO values and probability of Barlett’s sphericity test for questionnaires.

Name of questionnaire	KMO value	Significant probability of Barlett’s test sphericity
SCL-90	0.938	0.000
PSQ	0.897	0.000
NEO-FFI-N	0.783	0.000

Validity of the questionnaire mainly refers to construct validity which is the measured values explanation degree of psychological trait of participants. The construct validity of the questionnaire includes convergent validity and discriminant validity. In this study, composite reliability (CR) and average variance extracted (AVE), proposed by Chen et al. (2016), were applied to judge the goodness of convergent validity. In general, AVE > 0.5 or CR > 0.6 indicates high convergent validity. The AVE and CR values for each questionnaire used in this study are presented in Table 4. It can be seen that the CR values of the three scales are 0.973, 0.817, and 0.69, respectively. All the values are greater than 0.6, which meets the measurement requirements and indicates that the three questionnaires show internal convergent validity.

**TABLE 4:** Convergent validity analysis of the questionnaire.

Questionnaire name	AVE	CR
SCL-90	0.294	0.973
PSQ	0.242	0.796
NEO-FFI-N	0.193	0.69

In this study, the psychological symptom scale and the occupational strain scale are multi-dimensional and hence need to be tested for discriminant validity. The discriminant validity of these questionnaires is evaluated by calculating the square root of the AVE value. If the square root of the AVE value is greater than the correlation coefficient value of each dimension, the discriminant validity of the questionnaire is excellent. The diagonal values in Tables 5, 6 represent the square root of AVE values in SCL-90 and PSQ, respectively, and the other values represent the correlation coefficient values of each dimension. It can be seen from the tables that the square roots of the AVE values of each dimension in the scales are greater than the correlation coefficient values of each dimension; therefore, the discriminant validity of the selected questionnaires is excellent. From this analysis, the selected SCL-90 and PSQ scales are reliable and can be effectively applied for the survey analysis of metro drivers.

**TABLE 5:** Discriminant validity analysis of SCL-90.

	F1	F2	F3	F4	F5	F6	F7	F8	F9	F10
F1	0.592									
F2	0.635	0.692								
F3	0.51	0.744	0.817							
F4	0.697	0.815	0.755	0.807						
F5	0.673	0.753	0.719	0.826	0.837					
F6	0.603	0.671	0.6	0.7	0.703	0.745				
F7	0.526	0.64	0.681	0.724	0.711	0.581	0.74			
F8	0.596	0.713	0.744	0.774	0.739	0.669	0.654	0.79		
F9	0.63	0.752	0.776	0.815	0.816	0.694	0.699	0.794	0.845	
F10	0.661	0.659	0.56	0.7	0.675	0.565	0.532	0.624	0.646	0.717

**TABLE 6:** Discriminant validity analysis of PSQ.

	VS	PSY	IS	PHS
VS	0.519			
PSY	0.497	0.603		
IS	0.474	0.542	0.582	
PHS	0.427	0.613	0.499	0.632

### Analysis of the Assessment Result

Table 7 shows the evaluation results of psychological symptoms among the metro drivers surveyed by SCL-90. In the table, somatization, compulsion, interpersonal relationship, depression, anxiety, hostility, terror, crankiness, and psychopathy are selected as the independent variables, and the results are compared with the Chinese adult norm for the SCL-90 scale. The Chinese adult norm for SCL-90 is regarded as the average score obtained by a nationwide random SCL-90 questionnaire survey of Chinese adults that was conducted by Tang et al. (1999) through integrating different results of the SCL-90 survey published in Chinese academic journals from 1987 to 1997. Currently, the Chinese adult norm for SCL-90 has been widely applied to evaluate the mental health condition of populations of different occupations. From the table, it can be found that the scores of somatization, compulsion, hostility, and psychopathy are significantly higher than the Chinese adult norm (*p* < 0.01). This indicates that the work of metro drivers mainly affects somatization, and the nature of work can easily induce a nervous emotion in metro drivers, thus resulting in negative psychological symptoms, such as compulsion, hostility, and psychosis. The score for interpersonal relationships is similar to the Chinese adult norm. This means that the work of metro drivers has little influence on interpersonal relationships. The total score of the metro driver is also significantly higher than the Chinese adult norms (148.84 ± 42.66) (*p* < 0.01). This indicates that the psychological symptoms are not optimistic in metro drivers. It is suggested that metro drivers should strengthen physical exercise to improve their physical fitness. In addition, metro drivers should always adjust their mentality through cultivating hobbies or communicating with family and friends.

**TABLE 7:** Results of psychological symptom assessment in metro drivers surveyed by SCL-90.

Psychological symptom	Metro drivers (*n* = 396)	Chinese adult norm	*t*
Somatization	1.61 ± 0.56	1.37 ± 0.48	8.682***
Compulsion	1.96 ± 0.63	1.62 ± 0.58	10.685***
Interpersonal relationship	1.68 ± 0.52	1.65 ± 0.51	1.113
Depression	1.68 ± 0.56	1.50 ± 0.59	6.260***
Anxiety	1.58 ± 0.53	1.39 ± 0.43	7.179***
Hostility	1.64 ± 0.66	1.48 ± 0.56	4.876***
Terror	1.45 ± 0.51	1.23 ± 0.41	8.333***
Crankiness	1.58 ± 0.55	1.43 ± 0.57	5.576***
Psychopathy	1.49 ± 0.47	1.29 ± 0.42	8.218***
Total score	148.84 ± 42.66	129.96 ± 38.76	8.805***

t is the statistical value of the Student’s t-test; ***p < 0.001. All dimensions are converted into factor scores for the Student’s t-test, and the total score is the sum of the original scores of the questionnaire.

Table 8 gives the evaluation results of occupational strain among metro drivers includes vocational strain, psychological strain, interpersonal strain, and physical strain. The evaluation results are also compared with the Chinese adult norm for PSQ. The Chinese adult norm for PSQ was estimated by Yang et al. (2007) by surveying 4,278 different occupational populations in China. Chinese adult norm for PSQ has been widely applied to evaluate the occupational strain of different occupations. From the table, it can be found that the scores of vocational strain and physical strain are significantly higher than the Chinese adult norm (*p* < 0.01). This indicates that the work intensity of metro drivers is greater than that observed in other occupations, and long-term work has an adverse effect on their business capabilities and physical health. The psychological strain of metro drivers is also higher than the Chinese adult norm. This means that metro drivers get easily nervous during work. The total score of the metro driver is also significantly higher than the Chinese adult norm (104.17 ± 14.18) (*p* < 0.01). The results show that the individual adaptability of most metro drivers cannot help them achieve a good balance of the job content.

**TABLE 8:** Occupational strain assessment results for metro drivers from PSQ.

Occupational strain	Metro driver (*n* = 396)	Chinese adult norm	*t*
Vocational strain	24.37 ± 3.71	20.4 ± 5.2	21.248***
Psychologic strain	25.52 ± 5.37	23.8 ± 5.9	6.370***
Interpersonal strain	28.17 ± 3.81	25.6 ± 4.4	13.418***
Physical strain	26.12 ± 4.82	22.6 ± 5.6	14.516***
Total score	104.17 ± 14.18	92.5 ± 17.3	16.376***

t is the statistical value of the Student’s t-test; ***p < 0.001.

### Correlation Analysis

To determine the main factor that influences the mental health of metro drivers, the correlation among occupational strain, neuroticism, and psychological symptoms is investigated. Table 9 shows the correlation coefficient (*r*) of each dimension in the SCL-90, PSQ, and NEO-FFI-N. It can be found that the neuroticism and psychological symptoms of metro drivers are significantly correlated with their occupational strain (*AP* = 0.40, *FP* = 0.78, *p* < 0.01). The occupational strain of metro drivers is positively correlated with psychological symptoms (*AF* = 0.45, *p* < 0.01). Neuroticism is positively correlated with psychological symptoms (*AP* = 0.53, *p* < 0.01), and it is positively correlated with occupational strain (*FP* = 0.44, *p* < 0.01). It can also be observed from other correlation coefficients that the various dimensions in scales are also positively correlated with each other, with *r* from 0.10 to 0.93, and all *p* < 0.05. This result indicates that the psychological symptom of metro drivers is mainly affected by occupational strain and neuroticism, but their influence mechanism is not clear and needs to be further investigated.

**TABLE 9:** Correlation coefficients of each dimension in the SCL-90, PSQ, and NEO-FFI-N for metro drivers.

	A	B	C	D	E	F	G	H	I	J	K	L	M	N	O	P
A	1															
B	0.72**	1														
C	0.86**	0.50**	1													
D	0.77**	0.47**	0.54**	1												
E	0.82**	0.43**	0.61**	0.50**	1											
F	0.45**	0.27**	0.47**	0.24**	0.40**	1										
G	0.36**	0.25**	0.37**	0.10*	0.37**	0.79**	1									
H	0.37**	0.21**	0.38**	0.22**	0.33**	0.88**	0.63**	1								
I	0.38**	0.27**	0.38**	0.26**	0.30**	0.83**	0.51**	0.74**	1							
J	0.43**	0.26**	0.44**	0.24**	0.39**	0.93**	0.70**	0.82**	0.76**	1						
K	0.39**	0.26**	0.39**	0.20**	0.35**	0.90**	0.67**	0.75**	0.72**	0.83**	1					
L	0.33**	0.15**	0.41**	0.17**	0.25**	0.79**	0.60**	0.67**	0.60**	0.70**	0.70**	1				
M	0.33**	0.23**	0.35**	0.18**	0.25**	0.78**	0.53**	0.64**	0.68**	0.72**	0.71**	0.58**	1			
N	0.44**	0.27**	0.47**	0.29**	0.34**	0.85**	0.60**	0.71**	0.75**	0.77**	0.74**	0.67**	0.65**	1		
O	0.41**	0.26**	0.43**	0.23**	0.37**	0.90**	0.63**	0.75**	0.78**	0.82**	0.82**	0.69**	0.70**	0.79**	1	
P	0.40**	0.17**	0.41**	0.21**	0.43**	0.78**	0.66**	0.66**	0.56**	0.70**	0.68**	0.56**	0.53**	0.62**	0.65**	1

All dimensions were positively correlated (p < 0.05). A represents PSQ total score; B represents vocational strain; C represents psychologic strain; D represents interpersonal strain; E represents physical strain; F represents SCL-90 total score; G represents somatization; H represents compulsion; I represents interpersonal relationship; J represents depression; K represents anxiety; L represents hostility; M represents terror; N represents crankiness; O represents psychopathy; P represents neuroticism. **p < 0.01.

### Mediating Effect of Neuroticism Between Occupational Strain and Psychological Symptoms

In this study, in order to further find the influence path among neuroticism, occupational strain, and psychological symptom, a path structural equation model is established using Amos24.0 software (Rezapur-Shahkolai et al., 2020), as shown in Figure 1. The model includes two sub-models: sub-model A and sub-model B. Sub-model A is established to investigate the effect of occupational strain on the psychological symptoms of metro drivers, with occupational strain as a predictor variable and psychological symptom as a result variable; Sub-model B is established by adding neuroticism as an intermediary variable to investigate the indirect effect of occupational strain on the psychological symptom of metro drivers.

**FIGURE 1:** The principle of path structural equation model: (I) sub-model **(A)**; (II) sub-model **(B)**. The numbers listed in the figures are standardized path coefficients (β); continuous pathways are significant at *p* < 0.01.

Before performing correlation analysis, the path structural equation model must be validated. In general, the structural equation model can be validated by evaluating fit indices of chi-square to freedom ratio (χ^2^/df), the goodness-of-fit index (GIF), normed fit index (NFI), comparative fit index (CFI), Tucker-Lewis (TLI), relative goodness-of-fit indices (RFI), and root-mean-square error of approximation (RMSEA). If the fit indices are within the recommended values, the model is valid. Table 10 presents the model fitting index and the recommended values. From the table, it can be observed that each fitting index is within the recommended range, which indicates the data and the models are well fitted in all aspects.

**TABLE 10:** Model fitting index of occupational strain and neuroticism on psychological symptoms of metro drivers.

Model fitting index	χ^2^/df	GFI	NFI	CFI	TLI	RFI	RMSEA
Recommended value	<5	>0.9	>0.9	>0.9	>0.9	>0.9	<0.08
Sub model A	3.508	0.918	0.946	0.961	0.953	0.935	0.075
Sub model B	3.497	0.911	0.940	0.957	0.948	0.929	0.075

Figure 1 also gives the value of standardized coefficient β, which is used to explain the element path relationship in the model. The value of β > 0 indicates that the elements are positively correlated, and a larger value means a stronger correlation. From the β-value in sub-model A (β = 0.52, *p* < 0.01), we can conclude that the occupational stain is strongly associated with psychological symptoms. The level of occupational strain in metro drivers can positively predict their psychological symptoms, and high occupational strain causes severe psychological symptoms. From the β-value in sub-model B, it can be found that the occupational strain of metro drivers has a significant positive predictive effect on the neuroticism (β = 0.49, *p* < 0.01) and psychological symptom (β = 0.34, *p* < 0.01), and the neuroticism had a significantly positive predictive effect on psychological symptom (β = 0.38, *p* < 0.01). After adding neuroticism as an intermediary in sub-model B, the direct predictive effect of occupational strain on the psychological symptom of metro drivers is decreased from β = 0.52 to β = 0.34. This indicates that neuroticism has a mediating effect between occupational strain and psychological symptoms.

To verify whether the mediating effect of neuroticism between occupational strain and psychological symptoms is significant or not, bootstrapping analysis was used to construct confidence intervals, to verify the significance of the mediation effect through analyzing the scores of 5,000 duplicate samples from 396 samples. The scores need to be judged according to the 95% confidence interval obtained by the bootstrap method. The lower confidence interval (LLCI) and the upper confidence interval (ULCI) do not contain 0 or possess the same symbol, that is, both values are negative or positive. If it is positive, it means that the parameter is statistically significant at the 0.05 level. Otherwise, if it contains 0, or an opposite symbol, it means that the parameter is not significant. Table 11 presents the results of neuroticism mediating the effect between occupational strain and psychological symptoms. The bias-corrected confidence intervals for the indirect effect is not equal to 0 (*b* = 0.03, 95% CI [0.015, 0.030]), and the mediating effect value is 0.187, accounting for 34.89% of the total effect. The result indicates that the neuroticism of metro drivers has a partial mediating effect between the occupational strain and psychological symptoms.

**TABLE 11:** Results of neuroticism mediating effect between occupational strain and psychological symptoms.

	Effect	Boot SE	Boot LLCI	Boot ULCI	*p*
Direct effect	0.348	0.070	0.023	0.061	0.000
Indirect effect	0.187	0.030	0.015	0.030	0.000
Total effect	0.536	0.057	0.043	0.082	0.001

*Boot SE, Boot LLCI, and Boot ULCI refer to standard error, 95% confidence interval lower limit, and upper limit of indirect effect estimated by deviation-corrected percentile bootstrap method, respectively.*

## Discussion

In this study, we focus on the psychological symptoms among metro drivers from the angle of occupational strain and neuroticism. A total of 396 metro drivers from Kunming Rail Transit Operation Co., Ltd. in China were investigated through a questionnaire survey. SCL-90, PSQ, and NEO-FFI-N were applied to evaluate the psychological symptoms, occupational strain, and neuroticism in metro drivers, respectively. The surveyed data were analyzed by SPSS software, and based on the data, a path structural equation model was established to explore the correlation among occupational strain, psychological symptoms, and neuroticism. The main conclusions of this study are given in the following section.

First, the total scores for psychological symptoms (148.84 ± 42.66) determined by SCL-90 are significantly higher than the Chinese adult norm (129.96 ± 38.76) in metro drivers, especially for the scores of somatization, compulsion, depression, anxiety, hostility, terror, crankiness, and psychopathy, with all the symptoms having a *p-*value < 0.01. This result is similar to that reported by Ma et al. (2020). The total scores for occupational strain (104.17 ± 14.18) are also higher in metro drivers when compared to the scores of Chinese adult norm (92.5 ± 17.3), especially for the scores of vocational strain, psychological strain, interpersonal strain, and physical strain (all *p* < 0.01). The results indicate that the mental health status of metro drivers is not optimistic. The metro drivers are likely to cause serious safety issues under a long-term fear of operating errors, excessive tension, chronic anxiety, and diffuse anxiety. Repeated and monotonous operating procedures can easily lead to somatization, paranoia, and other psychopathological symptoms in metro drivers. The closed and narrow working environment can make the metro driver feel at a loss in the event of an emergency and take wrong decisions in a panic (Kim et al., 2013; Biglari et al., 2016; Jung et al., 2018; Cho et al., 2019).

Second, the occupational strain among metro drivers is significantly positively correlated with psychological symptoms (*p* < 0.05). That is, the higher the occupational strain for metro drivers, the more obvious the psychological symptom. Neuroticism in metro drivers is also significantly positively correlated with occupational strain and psychological symptoms (*p* < 0.05). These results indicate that the neuroticism in metro drivers can positively predict their mental health and occupational strain.

Finally, we found that neuroticism has a partial mediating effect between the occupational strain and psychological symptoms in metro drivers. The mediating effect is 0.187, accounting for 34.89% of the total effect. That is, occupational strain can directly affect the psychological symptoms of metro drivers, which can further affect their psychological symptoms through the indirect effects of neuroticism. This result indicates that the occupational strain along with high neuroticism is more likely to adversely affect the mental health of metro drivers. The worse an individual’s ability to cope with pressure, the easier it is to develop neuroticism (Kotov et al., 2010). When individuals with high neuroticism face tension and stress, the psychological reaction is more obvious, and the long-term occupational strain will lead to psychological problems, such as anxiety, depression, and paranoia. In the face of stimuli, individuals with high neuroticism are more likely to show strong emotional reactions, and their ability to cope with emotions is also poor. They tend to adopt negative cognition and wrong coping strategies to deal with stimulus events (e.g., avoidance, anxiety, etc.), which may further lead to anxiety, depression, and other adverse psychological emotions (Liu et al., 2019).

In summary, occupational strain and mental health are not optimistic among metro drivers. The metro operating companies need to pay more attention to these problems. Based on the mediating role of neuroticism between the occupational strain and psychological symptoms, metro operating companies can facilitate the development of positive and stable personality characteristics in metro drivers, enable them to cultivate an optimistic and rigorous working attitude, and eventually inhibit the influence of occupational strain on their mental health. But personality, which is the individual cognitive, emotional, and behavioral process of psychological conditions, can be changed and deceived. Therefore, the mediating effect of neuroticism between the occupational strain and psychological symptom is limited, and it cannot be regarded as a determinant factor that affects the mental health of metro drivers.

## Conclusion

In this study, the correlation among psychological symptoms, occupational strain, and neuroticism among metro drivers is investigated through a questionnaire survey. The SCL-90, PSQ, and NEO-FFI-N are applied to evaluate psychological symptoms, occupational strain, and neuroticism among the metro drivers, respectively. The reliability and validity of the survey data were verified by SPSS software. The results show that the data can be effectively used to explore the relationship between occupational strain, neuroticism, and psychological symptoms of metro drivers. Based on the data analysis, it is found that the mental health of metro drivers is lower than recommended in the Chinese adult norm, and the occupational strain, psychological symptoms, and neuroticism are significantly positively correlated in metro drivers. In particular, there exists a superposition of occupational strain and adverse psychological symptoms. In addition, a path structural equation model (SEM) is established in AMOS software to further analyze the relationship among occupational strain, psychological symptoms, and neuroticism. The result shows that the direct effect of occupational strain on psychological symptoms is significant, and that neuroticism plays a mediating effect between occupational strain and psychological symptoms. The study result can provide a theoretical foundation for the metro operating companies to optimize the workflow for metro drivers.

Since this study only investigated the metro drivers of Kunming Metro Operation Co., Ltd., the sample is single and unrepresentative, and the research is still insufficient. In the future, the sample size can be expanded to conduct investigation and research on subway enterprises in different regions and different management levels. Relevant intervention strategies will also be formulated at the organizational and individual levels to improve the safety level of subway operations.

## Data Availability Statement

The raw data supporting the conclusions of this article will be made available by the authors, without undue reservation.

## Ethics Statement

Ethical review and approval was not required for the study on human participants in accordance with the local legislation and institutional requirements. The patients/participants provided their written informed consent to participate in this study.

## Author Contributions

JH and YZ: conceptualization and writing of the original draft. JH and SQ: methodology. YZ: software. JH, YZ, and WL: formal analysis, writing, reviewing, and language modification. All authors have read and agreed to the publication of the manuscript.

## Conflict of Interest

WL was employed by the Kunming Rail Transit Operation Co., Ltd. The remaining authors declare that the research was conducted in the absence of any commercial or financial relationships that could be construed as a potential conflict of interest.

## Publisher’s Note

All claims expressed in this article are solely those of the authors and do not necessarily represent those of their affiliated organizations, or those of the publisher, the editors and the reviewers. Any product that may be evaluated in this article, or claim that may be made by its manufacturer, is not guaranteed or endorsed by the publisher.
